The article "Direct-Contact Low-Frequency Ultrasound and Pulse Lavage Eradicates Biofilms on Implant Materials In Vitro" was published in 2021. Journal: Evid Based Complement Alternat Med.

# Direct-Contact Low-Frequency Ultrasound and Pulse Lavage Eradicates Biofilms on Implant Materials In Vitro

**DOI:** 10.1155/2021/1562605

**Published:** 2021-08-30

**Authors:** Xiaoqing Wu, Xuanren Shi, Mingcong Chen, Xiaoyong Chen, Chi Zhang, Xiaonan Zhang, Jinyu Zhu

**Affiliations:** ^1^Department of Orthopaedics and Traumatology, Shenzhen University General Hospital, Shenzhen 518055, China; ^2^Department of Hematology and Oncology, Shenzhen University General Hospital, Shenzhen 518055, China; ^3^Department of Laboratory Medicine, Shenzhen University General Hospital, Shenzhen 518055, China; ^4^Guangdong Key Laboratory for Biomedical Measurements and Ultrasound Imaging, School of Biomedical Engineering, Health Science Center, Shenzhen University, Shenzhen 518060, China; ^5^Department of Orthopaedics, Southern University of Science and Technology Hospital, Shenzhen 518055, China

## Abstract

Pulse lavage (PL) debridement and ultrasound are both known to be the treatment of biofilm-related periprosthetic joint infection (PJI). However, the efficacy of these in combination is unknown in eradicating biofilm from the orthopaedic metal implant surface. This study was conducted to understand the efficacy of PL and ultrasound in combination in eradicating bacterial biofilms on titanium alloy in vitro. Biofilms of *Staphylococcus aureus* strains were grown on titanium alloy coupons for 24 h. Then, the coupons were taken to each treatment group: (i) debrided with PL, (ii) exposed to ultrasound, or (iii) exposed to both. An untreated biofilm was set as a control group. Viable plate count and confocal microscopy using live/dead staining was used to measure the amount of biofilm. Viable plate count showed an approximate two-log reduction in CFU/cm^2^ in PL alone, from an initial cell count on the mental surface of approximately 10^9^ CFU/cm^2^. The ultrasound caused an approximate seven-log reduction, and the combination group eradicated viable biofilm bacteria completely. Confocal imaging corroborated the CFU data. Our results indicate that PL and ultrasound both are remarkably in eradicating biofilm, and the combination of PL and ultrasound is more effective than alone in reducing biofilm.

## 1. Introduction

Periprosthetic joint infection (PJI) is one of the most dreaded complications in joint replacement surgery, which is associated with pain, prolonged hospital stays, multiple surgeries, functional incapacitation, and even mortality [1]. Although the incidence of PJI is below 1-2%, with increasing number of patients undergoing joint replacement surgery, more implant-associated infections could happen [2].

These infections include acute infections (within the first 4 weeks after implantation) and late infections, which can be derived from either a perioperative contamination of the joint or an hematogenous spreading of bacteria to the joint [3]. The incidence of pathogenic microorganisms depends on the origin and the time interval after the index surgery. *Staphylococcus aureus* is the most commonly isolated bacteria in acute PJI cases, while coagulase-negative *Staphylococcus* and *Streptococcus* are dominant in late infections and hematogenous infections, respectively [4–6].

The article "Direct-Contact Low-Frequency Ultrasound and Pulse Lavage Eradicates Biofilms on Implant Materials In Vitro" was published in 2021. Journal: Evid Based Complement Alternat Med.

Infections by *S. aureus* are characterized by rapid form biofilms [7]. Biofilms, aggregates of bacteria cells embedded in an extracellular polymeric substances (EPS) matrix, are fundamental with respect to the pathogenesis and persistence of PJIs which protect the dividing bacteria from the immune system, antibiotics, and even mechanical debridement [8–10]. Despite recent improvements in understanding in biofilm, clinical success in eradicating PJI through revision surgery remains poor, even in the early postoperative period [11–13].

For acute PJI, debridement, antibiotics, and implant retention (DAIR) have been increasingly used due to less invasion and lower cost in contrast to two-stage exchange of the device. However, DAIR have higher failure rate (16–57.4%) [14–16], and *S. aureus* PJI appears to have lower success rate than other organisms [17, 18]. Inadequate removal of biofilms during the debridement is regard as the major reason of DAIR failures. Many different debridement techniques in vitro have been used to mechanically disrupt and remove bacterial biofilm established on implant materials, such as iodine immersion, pulse lavage (PL), or even mechanical brushing. PL is a common method which mechanically disrupts and removes bacterial biofilm established on bone, soft tissue, and implant materials. However, some studies have found that PL is inadequate at removal of biofilm from the surface of implant materials in vivo [19, 20].

For the last decade, sonication has emerged and gradually becomes a practical and effective method to dislodge biofilm and the associated bacteria from the surface of the implant. It was found that the biofilm on the prosthesis surface could be removed by ultrasonic vibration after the PJI prosthesis was taken out; the bacteria in the biofilm could be released, so as to improve the positive rate of bacterial culture. Unfortunately, although ultrasound has destroyed the biofilm almost completely, residual bacterial viability could still be detected [21–23]. Recently, a direct-contact low-frequency ultrasound (DCLFU) device was introduced for the purpose of wound debridement [24]. Further investigation found that DCLFU is a promising method to treat biofilm infections [25]. Therefore, we assume whether DCLFU and PL in combination can act on the surface of prosthesis to remove the biofilm. Here, we extend the study to biofilms grown on titanium alloy coupons and compare the efficacy of eradicating *S. aureus* biofilms using PL alone, DCLFU alone, and the two treatments in combination. If it can completely remove the biofilm on the surface of prosthesis, it will greatly improve the success rate of DAIR, which is undoubtedly a great news for PJI patients.

The article "Direct-Contact Low-Frequency Ultrasound and Pulse Lavage Eradicates Biofilms on Implant Materials In Vitro" was published in 2021. Journal: Evid Based Complement Alternat Med.

## 2. Materials and Methods

### 2.1. Bacterial Strain

As previously described, a clinically isolated *S. aureus* strain was used in this study [19]. *S. aureus* strain was grown on tryptic soy agar (TSA) (Oxoid, Cambridge, UK). Then, representative colonies were picked and suspended in trypticase soy broth (TSB; Rishui Biotechnology, Qingdao, China), growing at 37°C overnight with agitation (200 rpm). Bacteria were harvested and resuspended in TSB, adjusted to a turbidity equivalent to that of a 1 McFarland standard and diluted 1 : 3000, achieving the final cell concentration of approximately 1 × 10^5^ CFU/ml.

### 2.2. Biofilm Production

The biofilm was cultivated according to previously described steps with some modifications [20]. Briefly, biofilms were grown on titanium alloy coupons (10 × 10 × 1 mm, roughness 0.47, Beijing AK Medical Co., Ltd.). The coupons were putted in the 24-well clear bottom microtiter plates (Corning, Inc, Corning, NY). Subsequently, 2 ml bacteria suspension was added to each well and incubated for 24 hours at 37°C, 5% CO_2_.

### 2.3. Debridement

Coupons were followed by either (i) debridement with PL, (ii) debridement with DCLFU, or (iii) both. 3 L of normal saline was taken to irrigate each coupon with PL irrigation set at the high setting (Five Continents, Ningbo, China). During the operation, the nozzle was kept upright with about 3 cm distance from the surface of the coupon. A single operator moved the nozzle over the entire surface of coupon randomly but in an equal fashion, which aimed to create the same conditions in the operating room. According to the manufacturer's instructions, we performed sonication treatment (Scientz, Ningbo, China) with the following parameters: frequency of 25 kHz, flow rate of 15 ml/min saline solution, and a processing time of 1 min. The DCLFU device wide hatch probe was placed 2 mm above the coupons. Experiments were performed in triplicate.

### 2.4. Viable Cell Count

After exposure to the treatments, phosphate buffered saline (PBS; Dulbecco's, Gibco, Grand Island, NY) were used to rinse each coupon. Sonicating for 15 min at a frequency of 35 kHz in the 10 ml of PBS was used to remove the biofilm. Totally, sonication was duplicated three times. Between each time, there is a 10 s vortex period. A 10-fold serial dilution was prepared and plated onto a solid agar, which were incubated for 24 h (37°C, 5% CO_2_), and then, the number of colony forming units (CFU) was counted, expressed as CFU/cm^2^.

The article "Direct-Contact Low-Frequency Ultrasound and Pulse Lavage Eradicates Biofilms on Implant Materials In Vitro" was published in 2021. Journal: Evid Based Complement Alternat Med.

### 2.5. Confocal Laser Scanning Microscopy (CLSM)

Confocal laser scanning microscopy (CLSM, Olympus FV10i, Waltham, MA) was used in the control group and treatment group to image the bacterial biofilms and conform the CFU data. The bacterial biofilms were observed using live-dead staining (Invitrogen Molecular Probes, USA) following the manufacturer's instructions. The Live-Dead kit contains SYTO-9 that stains viable bacterial DNA green, and dead cells appear red when propidium iodide (PI) enters compromised bacterial cell membranes. After exposure to the treatments, the coupons were lightly dipped in sterile water three times in order to remove nonfirmly attached bacteria and debris. Then staining for 15 min at room temperature in the dark, biofilms were rinsed with PBS to remove the extracellular dyes and observed with CLSM.

### 2.6. Statistical Analysis

CFU data were first log10 transformed. Statistical comparisons between the geometric means of CFU/cm^2^ from control and treatment groups were performed using SPSS Version 19 (IBM SPSS Statistics for Windows, Version 19.0 Armonk, NY: IBM Corp.) using an unpaired, two tailed Student's *t*-test assuming equal variance. Statistical significance was determined if *p* < 0.05.

## 3. Results

### 3.1. Viable Cell Count

In this study, the number of CFU on coupons aims to quantify bacteria. In the control group, the biofilms had grown to approximately 10^9^ CFU/cm^2^ after 24 h (Figure 1). In the treatment group, PL debridement showed an approximate two-log reduction in CFU/cm^2^ compared to the control group (*p* < 0.05), whereas exposure to DCLFU indicated an approximate seven-log reduction (*p* < 0.05). The bacteria cannot be detected in debridement PL and DCLFU exposure, which is accounting for a nine-log reduction (*p* < 0.05).

### 3.2. Confocal Microscopy

Confocal microscopy was a useful method which can measure the level of biofilm debrided following pulse lavage irrigation and DCLFU (Figure 2). After PL the biofilm cell density and viability had been reduced (Figure 2). The coupon exposed to DCLFU showed even more reduction of surface attached bacteria (Figure 2). The combination of PL and DCLFU showed the least cells remaining on the surface, and they were almost all dead (red) (Figure 2).

## 4. Discussion

With the formation of biofilms and bacterial growth, it results in a refractory infection of the implants. Since high risks of infection could occur perioperatively, there is an urgent need for a novel and effective way to remove bacterial biofilms from the implants. In this study, we investigated the effect of PL and DCLFU on eradication of biofilm formed by *S. aureus* on the titanium alloy surface.

The article "Direct-Contact Low-Frequency Ultrasound and Pulse Lavage Eradicates Biofilms on Implant Materials In Vitro" was published in 2021. Journal: Evid Based Complement Alternat Med.

PL irrigation is a commonly used technique for debridement. Our results showed that PL reduced bacterial colonization by approximately two log number of cells. CLSM also showed that the biofilm had been reduced to a monolayer of cells on the surface, and the remaining cells appeared to be mostly viable after PL. These findings are consistent with previous studies that reported approximately two-log reduction in cell numbers following PL [20, 26]. Knecht et al. [20] have demonstrated that PL reduced the CFU count of strain of biofilms by approximately two orders of magnitude, from an initial cell count on the metal surface of approximately 10^9^ CFU/cm^2^. These studies illustrate that PL irrigation of implant materials removed a substantial mass of biofilm. Besides, it is also found that a substantial mass of biofilm still remains. Furthermore, some authors have found that residual bacteria on the coupons after PL were sufficient to restore a biofilm after incubation [27]. Therefore, a new debridement method which can completely remove the biofilm is needed.

Low-frequency ultrasound is a promising method to treat biofilm infections due to its advantages, such as beam directivity and capability of treating deep tissue targets without tissue damage [28]. Previous studies have demonstrated the effectiveness of ultrasound in treating biofilms [29, 30]. In our study, DCLFU alone resulted in approximately seven log CFU/cm^2^ reduction of biofilm cells. CLSM show that there is a significant reduction in biofilm burden but not completely with regard to DCLFU alone. These findings were supported by some other studies. Singh et al. found that sonication treatment did not manage to destroy the biofilm completely [21]. Ensing et al. concluded that ultrasound alone did not negatively affect bacterial viability, neither in planktonic state nor in biofilm [31]. In contrast, Nishikawa et al. showed that *Staphylococcus* biofilm can be effectively removed by ultrasonic exposure in the animal model [32]. Granick et al. have demonstrated that the biofilm was cleared off completely from titanium and stainless steels implant materials when treated with DCLFU [25]. Numbers of factors could cause the observation bias. Such as the frequency, the configuration, the intensity, the exposure time, and the material, these are all important factors in consideration whether biofilms can be eradicated. However, there is growing evidence that ultrasonic treatment alone does not seem to be capable of completely eradicating biofilms on its own.

The article "Direct-Contact Low-Frequency Ultrasound and Pulse Lavage Eradicates Biofilms on Implant Materials In Vitro" was published in 2021. Journal: Evid Based Complement Alternat Med.

The combination of sonication with other technologies such as high pressure requires further investigations as pointed out in a review by Piyasena et al. [33]. To the best of our knowledge, it is the first time to investigate the effects of DCLFU in combination with PL against *S. aureus* biofilm in vitro. In the present study, reductions of approximately two log CFU/cm^2^ and seven log CFU/cm^2^, respectively, were observed with PL and DCLFU alone. When PL were combined with DCLFU, the reduction of cell increased, reaching proximately nine log CFU/cm^2^, implying a synergistic effect. The synergistic effect of PL and DCLFU remains unclear. It seems likely that PL reduces the load of bioburden, DCLFU mechanical destruction due to cavitation and acoustic microstreaming. It still needs to be clarified in future study.

There were some limitations in our study. First, we did not assess the implant surface modifications such as surface roughness, which significantly impacts on implant longevity [34]. Second, it may not be applicable to other types of bacteria, such as MRSA, because we used a single strain experimental model. Third, our study only focused on titanium alloy, and other materials of commonly used orthopaedic implants still need to be further investigated.

The present study provided insight into the elimination of biofilm formed by *S. aureus* on titanium alloy using PL or DCLFU alone or in combination. Our experimental evidence strongly indicated that that PL or DCLFU technique alone did not have the ability to completely eradicate the biofilms in our model system. Conversely, the combination could clear the biofilms off from the implant materials totally. Our results suggest that the combination of PL and DCLFU might be an optimal technique in debridement for infected total joint implants. It will improve the success rate of DAIR in the early PJI while to avoid two-stage reimplantation that would bring patients more costs and risks.

## Figures and Tables

**Figure 1:** Biofilm cell density quantified after treatment demonstrating a reduction in biofilm mass. C, control group; PL, pulse lavage group; DCLFU, direct-contact low-frequency ultrasound group; PL + DCLFU, combination of the PL and DCLFU group. ^*∗*^, ^*∗∗*^, and ^*∗∗∗*^ indicate statistically significant log reductions compared to successive groups.

**Figure 2:** Confocal laser scanning microscopic images showing *S. aureus* of control, pulse lavage (PL), and direct-contact low-frequency ultrasound (DCLFU) treatment groups. Live cells are stained green (appears bright in grayscale) and dead cells are strained red (appears dim in grayscale). The scale bar represents 100 *μ*m magnification.

The article "Direct-Contact Low-Frequency Ultrasound and Pulse Lavage Eradicates Biofilms on Implant Materials In Vitro" was published in 2021. Journal: Evid Based Complement Alternat Med.

## Data Availability

The data generated or used to support the findings of this study are included within the article.
